# Image Enhancement Algorithm-Based Ultrasound on Pelvic Floor Rehabilitation Training in Preventing Postpartum Female Pelvic Floor Dysfunction

**DOI:** 10.1155/2022/8002055

**Published:** 2022-04-19

**Authors:** Lifeng Chen, Chunyan Lu

**Affiliations:** ^1^Department of Urology, Affiliated Xiaoshan Hospital, Hangzhou Normal University, Hangzhou, 311200 Zhejiang, China; ^2^Department of Operating Room, Affiliated Xiaoshan Hospital, Hangzhou Normal University, Hangzhou, 311200 Zhejiang, China

## Abstract

In order to explore the application value of image enhancement algorithm in evaluating pelvic floor rehabilitation training in the prevention of postpartum female pelvic floor dysfunction (FPFD), 70 patients with FPFD were selected as the study subjects and randomly divided into two groups. One group received routine nursing (control group, *n* = 35), and the other group received pelvic floor rehabilitation training based on routine nursing (experimental group, *n* = 35). In ultrasound images based on an image enhancement algorithm, the International Consultation on Incontinence Questionnaire-Short Form (ICIQ-SF), and Pelvic Floor Distress Inventory-20 (PFDI-20) were used to evaluate the efficacy. The results showed that after image enhancement algorithm processing, the image signal-to-noise ratio (SNR), peak signal-to-noise ratio (PSNR), and structural similarity index (SSIM) of ultrasound images of patients with FPFD were significantly improved (*P* < 0.05); the mean square error (MSE) was significantly decreased (*P* < 0.05); the diagnostic accuracy of FPFD in the original ultrasound images was 73.34%, and that after image enhancement algorithm processing was significantly improved to be 89.86% (*P* < 0.05). In addition, the overall clinical response rate of FPFD in the experimental group (82.86%) was obviously higher than that in the control group (51.43%) (*P* < 0.05). After rehabilitation training, the ICIQ-SF and PFDI-20 scores of patients with FPFD in the two groups suggested a significant decrease (*P* < 0.05). In summary, using an image enhancement algorithm has a good application prospect in evaluating pelvic floor rehabilitation training in preventing postpartum FPFD and is worthy of further promotion.

## 1. Introduction

Female pelvic floor dysfunction (FPFD) is a group of diseases mainly caused by defects, degeneration, injury, and dysfunction of pelvic support structures, and stress urinary incontinence, pelvic organ prolapse, sexual dysfunction, chronic pelvic pain, and fecal incontinence are common, which seriously affect women's quality of life [1–3]. FPFD is caused by pelvic floor muscle injury due to pregnancy, delivery, aging, obesity, cough, constipation, and other reasons, which in turn affects the function of pelvic floor bracketing [4]. At present, in the process of clinical FPFD diagnosis, commonly used imaging methods include intracavitary ultrasound, tomographic ultrasound imaging, dynamic pelvic floor MRI, and intracavitary MRI [5, 6].

Pelvic floor rehabilitation training is a relatively rapidly developing rehabilitation field in recent years. It is a rehabilitation training method to promote the recovery of nerves and muscles injured during pregnancy and delivery, which can improve the long-term pelvic floor conditions, while reducing the chance of FPFD due to changes in anatomical structure and age [7–10]. Studies have shown that pelvic floor training during pregnancy can reduce the incidence of FPFD in primipara 3 months after delivery, and postpartum rehabilitation can significantly reduce the incidence of FPFD 6-12 months after delivery [11–13]. The postpartum period is a favorable period for the prevention and treatment of FPFD. At present, the main pelvic floor rehabilitation training methods include biofeedback and electrical stimulation therapy [14]. Electrical stimulation therapy is to achieve the purpose of exercise by giving muscle electrical stimulation and allowing it to contract passively; biofeedback is to accelerate the speed of rehabilitation by actively performing contractile muscle exercise. Sometimes, the combination of electrical stimulation therapy and biofeedback can also be used to achieve better pelvic floor muscle rehabilitation training effect [15, 16].

At present, there have been many reports on the study of ultrasound image diagnosis for postpartum female patients with FPFD, and there are endless studies on pelvic floor rehabilitation for this type of disease [17]. Pelvic floor ultrasound is a commonly used clinical imaging method. It can help evaluate the degree of FPFD, find out the damage and degree of levator ani and anal sphincter muscle, and be used for postoperative observation of pelvic floor surgery. It is suitable for urinary incontinence, pelvic organ prolapses, fecal incontinence, and other diseases. However, there is no study on the image enhancement algorithm for ultrasound image characteristics of patients with FPFD, while there is no report on the relevant studies on the ultrasound image enhancement algorithm for FPFD. Therefore, it hopes to design an image enhancement algorithm for the ultrasound image characteristics of patients with FPFD and use it in the ultrasound image diagnosis process of pelvic floor rehabilitation training effect for clinical patients with FPFD. Evaluating the algorithm performance and comparing the diagnostic accuracy are performed to comprehensively assess the application potential of this algorithm and the efficacy of pelvic floor rehabilitation training in the prevention of FPFD.

## 2. Materials and Methods

### 2.1. Study Subjects

Seventy patients with FPFD diagnosed in hospital from February 2018 to February 2021 were selected as the study subjects, and all patients underwent intracavitary ultrasonography. The age range of the patients was 33-76 years; the mean age was 48.48 ± 7.29 years. The following is the prevalence of all patients: 22 patients with pelvic floor organ prolapse, 31 patients with urinary incontinence, and 17 patients with bulging posterior vaginal wall. All procedures of this study had been approved by the ethics committee of hospital, and all subjects signed the informed consent form.

The following are the inclusion criteria: patients diagnosed with FPFD and patients who had signed informed consent. The following are the exclusion criteria: patients with severe renal disease or other organic diseases, patients in lactation, and patients in pregnancy.

### 2.2. Nursing and Rehabilitation Training Methods

According to the method of digital random grouping, all patients were divided into two groups, with 35 cases in each group. One group was given routine nursing, which was recorded as the control group. Another group added pelvic floor rehabilitation training based on routine nursing. Pelvic floor rehabilitation training included pelvic floor muscle training and pelvic floor biofeedback training. Pelvic floor muscle training was carried out by placing a vaginal dumbbell in the vagina once a day for 15 minutes each time. Pelvic floor biofeedback training was carried out through the pelvic floor rehabilitation therapeutic apparatus; the treatment frequency was twice a week, 20 minutes each time.

### 2.3. Ultrasound Examination of Pelvic Floor

Voluson E8 color Doppler ultrasound system (GE, USA) was used. Pelvic floor ultrasonography was performed in both groups. The probe was used to scan the vagina, urethra, and bladder neck of the subjects at rest and contraction, and the angle between the middle line of pubic symphysis and the lower edge of pubic symphysis line to the bladder neck and the movement angle of the bladder neck were measured.

### 2.4. Establishment of Ultrasonic Image Optimization Model for Patients with FPFD Based on Image Enhancement Algorithm

Using the advantages of fast operation speed and good noise reduction effect of median filtering algorithm, combined with the architecture of adaptive median filtering and the idea of pixel classification, an adaptive median filtering algorithm for pelvic floor ultrasound is designed. Firstly, the gray value is set up as *F*(*a*, *b*), and then an ascending array is established, which includes the gray values of *F*(*a*, *b*) and other pixels in its neighborhood. The positions of the minimum, maximum, median, maximum nonminimum, and minimum nonmaximum of the ascending array are represented as *S*_min_, *S*_max_, *S*_med_, *S*[*N*1], and *S*[*N*2]. Then, with a fixed size of the filter window (taking 3 × 3 window as an example) as the interval, the size relationship between the current pixel and the extreme point is compared. If the median *S*_*med*_ of the filter window is not noise and the current pixel is the extreme point of the filter window, it is determined as a quasi-noise point (it needs to be determined twice); otherwise, it is determined as a signal point (no processing).

If the current point is the minimum value, the slope *K*1 selects the slope from point *N*1 to the middle point of all minimum values to represent the slope in the neighborhood of the current point (Equation (1)); the slope *K*2 is the slope from *N*1 to *N*2, which is used to represent the average slope of the entire filtering window (Equation (2)); if the current point is maximum, the slope *K*1 selects the slope from point *N*1 to the midpoint of all maximums to represent the slope in the neighborhood of the current point (Equation (3)); the slope *K*2 is the slope from *N*1 to *N*2, which is adopted to denote the average slope of the entire filtering window (Equation (4)).

(1) $$\begin{array}{c} K1=\frac{S\left[N1\right]-F\left(a,b\right)}{\left(N1+1\right)/2}, \end{array}$$

(2) $$\begin{array}{c} K2=\frac{S\left[N2\right]-S\left[N1\right]}{\left(N2-N1\right)}, \end{array}$$

(3) $$\begin{array}{c} K1=\frac{F\left(a,b\right)-S\left[N1\right]}{\left[M\times \left(M-1\right)-N2\right]}, \end{array}$$

(4) $$\begin{array}{c} K2=\frac{S\left[N2\right]-S\left[N1\right]}{\left(N2-N1\right)}. \end{array}$$

After the preliminary screening of the quasi-noise points, the threshold *Q* is used for the second determination. The threshold is expressed in

(5) $$\begin{array}{c} Q=\frac{S_{\text{med}}}{\varepsilon }. \end{array}$$

*S*_*med*_ represents the median of the filter window, and *ε* means the positive integer. The threshold is adaptively selected according to *S*_*med*_ when judging the quasi-noise point, and the *ε* value determines the threshold. The same peak signal-to-noise ratio (PSNR) and mean square error (MSE) are also affected by the *ε* value.

On this basis, it introduces the morphological gradient operator to effectively identify and enhance the edge image (set as *P*) of the pelvic floor ultrasonic image. Based on the existing antinoise expansion gradient operator (Equation (6)), antinoise corrosion gradient operator (Equation (7)), and antinoise expansion corrosion gradient operator (Equation (8)) [18], two improved gradient operators are designed for edge detection of pelvic ultrasound image according to the characteristics of ultrasonic image and the properties of each operation of gray morphology. The expressions are shown in Equations (9) and (10).

(6) $$\begin{array}{c} P_{1}\left(g\right)=g⊕D-g\cdot D, \end{array}$$

(7) $$\begin{array}{c} P_{2}\left(g\right)=g\circ D-g\Theta D, \end{array}$$

(8) $$\begin{array}{c} P_{3}\left(g\right)=\left(g\circ D\right)⊕D-\left(g\cdot D\right)\Theta D, \end{array}$$

(9) $$\begin{array}{c} P_{4}\left(g\right)=\left(g\circ D\right)⊕D-g\circ D, \end{array}$$

(10) $$\begin{array}{c} P_{5}\left(g\right)=g\cdot D-\left(g\cdot D\right)\Theta D. \end{array}$$

*g* denotes the input image, and *D* represents the structural elements. The algorithm first obtains the edge image of the ultrasonic image through the morphological gradient operator and then enhances the edge region corresponding to the original image, and the nonedge region remains unchanged, so as to achieve the overall image enhancement effect of the pelvic floor ultrasonic image of patients.

### 2.5. Evaluation of Pelvic Ultrasonic Image Quality Based on Image Enhancement Algorithm

The image signal-to-noise ratio (SNR), PSNR, MSE, and structural similarity index (SSIM) [19] were used to measure the enhancement effect of pelvic ultrasound image and the maintenance of image edge area, and then, the application value of the algorithm was evaluated. The calculations of SNR, PSNR, MSE, and SSIM are shown in Equations (11), (12), (13), and (14), respectively.

(11) SNRri,rj=10×log∑p−1Grip−μri2∑p−1Grip−rjp210,

(12) PSNRri,rj=10×logGmax2∑p−1Grip−rjp210,

(13) $$\begin{array}{c} \text{MSE}\left(r_{i},r_{j}\right)=\frac{\sum_{p-1}^{G}r_{i}\left(p\right)-r_{j}{\left(p\right)}^{2}}{G}, \end{array}$$

(14) $$\begin{array}{c} \text{SSIM}\left(r_{i},r_{j}\right)=\frac{2\mu \left(r_{i}\right)\mu \left(r_{j}\right)+c_{1}}{\mu^{2}\left(r_{i}\right)+\mu^{2}\left(r_{j}\right)+c_{1}}\cdot \frac{2\sigma \left(r_{i}\right)\sigma \left(r_{j}\right)+c_{2}}{\sigma^{2}\left(r_{i}\right)+\sigma^{2}\left(r_{j}\right)+c_{2}}\cdot \frac{\mathrm{cov}\left(r_{i},r_{j}\right)+c_{3}}{\sigma \left(r_{i}\right)\sigma \left(r_{j}\right)+c_{3}}. \end{array}$$

*G* is the number of pixels in each image, and *μ*(*r*_*i*_), *μ*(*r*_*j*_), *σ*(*r*_*i*_), *σ*(*r*_*j*_) are the mean and variance of the image *r*_*i*_ and the image *r*_*j*_, respectively. cov(*r*_*i*_, *r*_*j*_) is the covariance of the image *r*_*i*_ and the image *r*_*j*_, *G*_max_ represents the maximum pixel value that each pixel in the image may obtain, and *c*_1_, *c*_2_, *c*_3_ are different parameters.

### 2.6. Observation Indicators of Rehabilitation Training Effect and Analysis of Imaging Diagnosis Effect

The International Consultation on Incontinence Questionnaire-Short Form (ICIQ-SF) and Pelvic Floor Distress Inventory-20 (PFDI-20) [20] were used to assess the recovery of urinary incontinence and quality of life of patients before and after pelvic floor rehabilitation training. Among them, the ICIQ-SF contains 3 items and 8 problems related to urinary incontinence, with a total score of 21 points. The higher the score, the more severe the urinary incontinence. The PFDI-20 contains 25 items, with a total score of 300 points. The higher the score, the worse the quality of life. The efficacy evaluation criteria for FPFD are given in Table 1.

### 2.7. Statistical Methods

The test data were processed by SPSS 19.0 statistical software. The measurement data were expressed as the mean ± standard deviation ($\overset{¯}{x}\pm s$). The comparison of mean between groups was performed by a *t* test. The enumeration data were expressed as percentage (%). The *χ*^2^ test was adopted. The differences were statistically significant when *P* < 0.05.

## 3. Results

### 3.1. Basic Information of Patients

Figure 1 indicates the comparison of the basic situation of the two groups of patients. There was no significant distinction between the mean age and mean disease duration of the two groups (*P* > 0.05); there was also no significant distinction between the number of types of FPFD in the two groups (*P* > 0.05).

### 3.2. Test Results of Ultrasonic Image Quality Based on Image Enhancement Algorithm

Figure 2 suggests the comparison of ultrasound image quality test results of patients with FPFD before and after image enhancement algorithm processing. After processing by the image enhancement algorithm, the SNR, PSNR, and SSIM of the ultrasound images of patients with FPFD were obviously improved (*P* < 0.05), and the MSE was clearly decreased (*P* < 0.05).

### 3.3. Ultrasound Image Analysis of Patients with FPFD Based on Image Enhancement Algorithm

Figure 3 is a comparative map of ultrasound images of patients with FPFD before and after algorithm processing. After the image enhancement algorithm processing, the ultrasound image of patients with FPFD achieved image enhancement while well maintaining the original shape of the edge region of the ultrasound image.

### 3.4. Evaluation of Rehabilitation Training Effect of Patients in the Two Groups

Figure 4 indicates the comparison of clinical efficacy between the two groups, and Figure 5 shows the comparison of ICIQ-SF and PFDI-20 scores between the two groups. The overall clinical response rate of FPFD in the experimental group was significantly higher than that in the control group, with statistical significance (*P* < 0.05). There was no significant difference in the ICIQ-SF and PFDI-20 scores between the two groups before rehabilitation training (*P* > 0.05), while the ICIQ-SF and PFDI-20 scores of the two groups of patients with FPFD showed a significant decrease after rehabilitation training (*P* < 0.05). The decrease in both scores in the experimental group was greater than that in the control group.

### 3.5. Ultrasound Image Diagnostic Evaluation of Pelvic Floor Rehabilitation Training

Figure 6 is a comparison of the diagnostic accuracy of ultrasound before and after image enhancement algorithm processing. The diagnostic accuracy of FPFD diseases in the original ultrasound image is 73.34%, and the diagnostic accuracy after image enhancement algorithm processing is 89.86%, which is significantly improved (*P* < 0.05).

## 4. Discussion

At present, in developed countries and regions such as Europe, America, Japan, and South Korea, pelvic floor rehabilitation training for postpartum female pelvic floor function has been quite popular, including pelvic floor muscle evaluation, biofeedback training, and electrical stimulation therapy [21]. Through this rehabilitation training, the nerves and muscles of the pelvic floor in patients with FPFD such as pelvic organ prolapse and urinary incontinence can be awakened, the vagina can be better restored to a tightened state, and the recovery of postpartum vaginal and pelvic floor muscle tension and elasticity can be accelerated. There were 70 patients with FPFD who were diagnosed in the hospital from February 2018 to February 2021 as the research objects. All the patients underwent intracavitary ultrasonography and were divided with 35 cases in the control group (routine nursing) and 35 cases in the experimental group (routine nursing+pelvic floor rehabilitation training) according to different nursing programs. First, the basic information of the two groups of patients were analyzed, from which no significant difference was found in the mean age, mean course of disease, and the number of FPFD types between two groups (*P* > 0.05). This provided a feasibility for follow-up research.

It compared the pelvic floor function recovery of patients with FPFD after conventional rehabilitation training and pelvic floor rehabilitation training intervention It was found that the overall clinical response rate of FPFD in the experimental group was significantly higher than that in the control group, with statistical significance (*P* < 0.05). This is similar to the research results of Jha et al. [22], indicating that pelvic floor rehabilitation training combined with routine nursing can highly improve the recovery efficiency of postoperative pelvic floor function, and the effect is better than that of single routine nursing. Figure 6 reveals that there was no significant difference in the ICIQ-SF and PFDI-20 scores between the two groups before rehabilitation training (*P* > 0.05), while the ICIQ-SF and PFDI-20 scores of the two groups of patients with FPFD showed a significant decrease after rehabilitation training (*P* < 0.05). The decrease in both scores in the experimental group was greater than that in the control group. It suggests that pelvic floor rehabilitation training has a significant effect on the recovery of pelvic floor function in patients with FPFD, which is consistent with the findings of Hagen et al. [23]. In addition, the gradient operator edge image enhancement algorithm has a good image enhancement effect on ultrasound images of patients with FPFD. The results showed that the SNR, PSNR, and SSIM of ultrasound images in patients with FPFD were significantly increased (*P* < 0.05), and the MSE was significantly decreased (*P* < 0.05). Compared with the original ultrasound image, the diagnostic accuracy of ultrasound image processed by the image enhancement algorithm was significantly improved (89.86%) (*P* < 0.05). Thus, it indicates that the gradient operator edge image enhancement algorithm has a good application prospect in the field of ultrasonic image enhancement.

## 5. Conclusion

According to the characteristics of pelvic floor ultrasound images in patients with FPFD, a gradient operator edge image enhancement algorithm was designed and used for ultrasound image evaluation of the effect of pelvic floor rehabilitation training in patients with clinical FPFD. The results revealed that ultrasound images based on an image enhancement algorithm could well evaluate pelvic floor rehabilitation training and significantly enhance the clinical diagnostic rate. However, there are some shortcomings; for example, the image enhancement algorithm remains to be optimized, and the efficacy evaluation indicators of pelvic floor rehabilitation training remain to be expanded. In conclusion, pelvic floor rehabilitation training can significantly improve the clinical symptoms of patients with FPFD, and ultrasound images based on image enhancement algorithm can significantly improve the clinical diagnostic accuracy of patients with FPFD, which has certain reference value for improving the clinical diagnosis and treatment efficiency of patients with FPFD.

## Figures and Tables

**Figure 1:** Comparison of basic information between the two groups. (a), (b), and (c) refer to pelvic floor organ prolapse, urinary incontinence, and bulging posterior vaginal wall, respectively.

**Figure 2:** Comparison of ultrasonic image quality test results of patients with FPFD before and after image enhancement algorithm processing. (a), (b), (c), and (d) are the contrast maps of SNR, PSNR, MSE, and SSIM values of ultrasound images of patients with FPFD before and after image enhancement algorithm processing, respectively; ∗ indicates that the differences are statistically significant compared with those before algorithm processing (*P* < 0.05).

**Figure 3:** Comparison of ultrasound images of patients with FPFD before and after algorithm processing. (a) and (c) are the ultrasound images of the experimental group before algorithm processing. (e) and (g) are the ultrasound images of the control group before algorithm processing. (b) and (d) are the ultrasound images of the experimental group after algorithm processing. (f) and (h) are the ultrasound images of the control group after algorithm processing, respectively.

**Figure 4:** Comparison of clinical efficacy between the two groups. (a) Comparison of efficacy; (b) comparison of overall response rate; ∗ indicates significant difference from the control group (*P* < 0.05).

**Figure 5:** Comparison of ICIQ-SF and PFDI-20 scores between the two groups. (a) ICIQ-SF score comparison diagram; (b) PFDI-20 score comparison diagram; ∗ means that there is a significant difference between ICIQ-SF score and PFDI-20 score or between the experimental group and the control group (*P* < 0.05).

**Figure 6:** Comparison of imaging diagnostic accuracy of different algorithms. ∗ indicates significant difference in diagnostic accuracy compared with original ultrasonic image (*P* < 0.05).

**Table 1:** Efficacy evaluation criteria for FPFD.

Curative effect	Symptoms	Pelvic floor muscle strength
Significantly effective	Symptoms disappear	>grade 3
Effective	Symptoms and pelvic floor function improved	Grades 2~3
Ineffective	Symptoms and pelvic floor function unchanged or worsened	<grade 2

## Data Availability

The data used to support the findings of this study are available from the corresponding author upon request.
